# CYPA promotes the progression and metastasis of serous ovarian cancer (SOC) in vitro and in vivo

This article has been retracted.

**DOI:** 10.1186/s13048-019-0593-2

**Published:** 2019-11-29

**Authors:** Zhi-Ying Qi, Fang Wang, Ying-Ying Yue, Xue-Wang Guo, Rui-Meng Guo, Hong-Lin Li, Yan-Ying Xu

**Affiliations:** Department of gynecolog, the second hospital of Tianjin medical university, No.23 Pingjiang road, Hexi district, Tianjin, 300211 China

**Keywords:** Serous ovarian cancer (SOC), CYPA, Migration, Invasion, Therapeutic target

## Abstract

Ovarian cancer (OC) is a type of gynaecological malignancy with high mortality in females. Serous ovarian cancer (SOC) is a distinct subtype of OC with poor early diagnosis. Given the limitations of traditional therapies, such as chemotherapy, targeted treatment is therefore a promising therapy to improve the survival rate of SOC patients. Cyclophilin A (CYPA) is a member of Cyclophilin family and thought to participates in multiple cellular processes such as cell transduction and immune modulation. Recently, various of studies indicated that CYPA has critical impact on cancer progression. CYPA could regulate cell proliferation, invasion, and chemoresistance of multiple types of cancers. However, it is still unclear whether it could affect ovarian cancer. In this study, we demonstrated that CYPA was highly expressed in SOC tissues compared with adjacent tissues. Further, CYPA was significantly associated with clinical stage and lymphnode metastasis of SOC patients. Additionally, data indicated that knockdown of CYPA by its shRNA dramatically reduces migration and invasion capacity of SOC cells in vitro and blocks tumor metastasis in vivo. Our study investigates the involvement of CYPA in the progression and metastasis of SOC, and therefore provides CYPA as a promising therapeutic target for SOC treatment.

## Introduction

Ovarian cancer (OC) is s the seventh most common cancer and a type of gynaecological malignancies, with high mortality in females [1–3]. The majority of ovarian cancers (nearly 90%) are originated from epithelial tissues [4, 5]. Despite ongoing efforts to find effective treatment methods for OC, the overall survival rate remains less than 30%, which was mainly caused by the difficulty for early diagnosis, and often results in a poor prognosis [6, 7]. Serous ovarian cancer (SOC) is a distinct histological subtype of OC, which is usually diagnosed at advanced stage [8]. Although chemotherapy is the established treatment for SOC, the survival rate remains low, and it is highly anticipated that new treatments will be successfully developed [9, 10]. Therapies, such as targeted treatment and immunotherapy, are needed to combat this disease [11, 12]. Recently, various of proteins have been found highly expressed in SOC tissues, some of which (including AIF1 and WNK1) have become potential therapeutic targets for SOC [13]. To improve the prognosis of SOC patients, novel therapeutic targets are still needed to be developed.

Cyclophilins are a class of highly conserved cellular proteins, which have specific chemical structures containing 109 amino acids and could interact with other proteins from different locations and of multiple functions [14, 15]. Previous reports indicated the main functions of cyclophilins was protein folding and trafficking [16]. Cyclophilin A (CYPA), which has the capacity to bind the immunosuppressive drug cyclosporin A (CSA), was first purified from bovine thymocytes [17]. CYPA is thought to play critical roles in many cellular processes, such as cell transduction and immune modulation [18]. Additionally, CYPA could interact with the matrix protein of influenza A virus so that to restrict virus replication [19], and the concentration of CYPA in serum was obviously correlated with the prognosis after hemorrhagic stroke [20]. Notably, more and more studies indicated that CYPA has critical impact on cancer progression.

CYPA is widely expressed in normal tissues and highly expressed in various tumors, such as non small cell lung cancer (NSCLC) and pancreatic cancer [21]. Previous studies demonstrated that CYPA could regulate cell proliferation, invasion, apoptosis, and chemoresistance of multiple types of cancers [22, 23]. For an example, a previous study showed that CYPA could interact with CD147, thereby promoting cell proliferation of pancreatic cancer [24]. Although CYPA plays an important role in tumorigenesis, it is still unclear whether it could participate in the progression of ovarian cancer.

Interestingly, we found the high expression of CYPA in human SOC tissues and analyzed the potential link between CYPA expression and clinical features of SOC patients. We also revealed that CYPA depletion dramatically blocked SOC cell migration and invasion and further suppressed tumor metastasis in mice. Therefore, CYPA could serve as a potential therapeutic target for SOC treatment.

## Materials and methods

### Antibodies, primers and shRNA plasmids

Anti- Cyclophilin A (CYPA) antibody (for immunohistochemicstry, 1:100 dilution, for immunoblot, 1:1000 dilution, #ab154388, Abcam, Cambridge, UK), Anti-β-actin (1:1000 dilution, #ab8226, Abcam, Cambridge, UK). Anti-MMP3 antibody (1:500 dilution, #ab52915, Abcam, Cambridge, UK), Anti-MMP9 antibody (1:1000 dilution, #ab38898, Abcam, Cambridge, UK).

The quantitative RT-PCR primer sequences of CYPA were as follows: forward,5′ - GGTCCTGGCATCTTGTCCAT-3’ and reverse, 5′- AACACCACATGCTTGCCATC-3′; The quantitative RT-PCR primer sequences of GAPDH were as follows: forward, 5′- CGACCACTTTGTCAAGCTCA − 3′ and reverse, 5′- GGTTGAGCACAGGGTACTTTATT-3′.

Ready-to-package AAV shRNA clone for CYPA was purchased from Addgene, and the targeted sequences of CYPA were as follows: 5′ - CCTTTGAGCTGTTTGCAGACAAG − 3′.

### Human tissue samples and analysis

Human SOC tissues and adjacent tissues were collected from the patients receiving surgical treatment in the second hospital of Tianjin medical university. Mice tumor tissues taken were isolated from mice in the metastasis assays.

The clinical features, including patient age, tumor size, preoperative chemotherapy, tumor differentiation, International Federation of Gynecology and Obstetrics (FIGO) stage and lymphnode metastasis were recorded and listed in Table 1.

**Table 1:** Relationships of CYPA and clinicopathological characteristics in 82 patients with tongue squamous cell carcinoma

Feature	All *n* = 82	CYPA expression		χ^2^	P
		Low	High		
		*n* = 42	*n* = 40		
Age (year)				0.532	0.466
< 55	50	24	26		
≥ 55	32	18	14		
Tumor size				1.717	0.190
< 10 cm	45	26	19		
≥ 10 cm	37	16	21		
Preoperative chemotherapy				2.513	0.113
Yes	36	22	14		
No	46	20	26		
Differentiation				3.241	0.072
Low	24	16	8		
High	58	26	32		
FIGO stage				4.228	0.040*
I-II	34	22	12		
III-IV	48	20	28		
Lymphnode metastasis				5.859	0.015*
Yes	38	14	24		
No	44	28	16		

*p < 0.05

To explore the possible relation between the expression level of CYPA and SOC progression, immunohistochemistry (IHC) assays were performed. Briefly, sample sections were fixed with 4% PFA for 30 min and subsequently blocked with 2% BSA for 20 min. Slides were incubated with CYPA, MMP3, MMP9 antibodies at room temperature for 2 h. Subsequently the sections were incubated with biotinylated secondary antibody for 1.5 h, and diaminobenzidine was used as a chromogen substrate.

CYPA was found mainly located in the cytoplasm of SOC tissues. The score method was as follows. Briefly, the proportion of positive stained cells was graded as follows: 0, negative cells; 1, 10–50% positive cells and 2, > 50% positive cells. The staining intensity was evaluated on a score of 0 (no staining), 1 (modest staining) and 2 (strong staining). The expression level of CYPA was measured based on the staining index: staining intensity score + positive tumor cell staining score. Staining index 0, 1, 2 was considered relatively low expression, while staining index 3 and 4 was considered high expression.

### Cell culture and transfection

CAOV3 and OVCAR3 human SOC cells were bought from American Type Culture Collection (ATCC, Manassas, VA). CAOV3 and OVCAR3 cells were maintained in DMEM or RPMI-1640 culture medium, respectively, and supplemented with 10% of fetal bovine serum (FBS, Gibico, Grand Island, NY, USA Bio-Rad, CA, USA). Cells were maintained at 37 °C in a 5% CO_2_ incubator.

The plasmids of CYPA shRNA were transfected into SOC cells using lipofectamine 2000 (#11668019, Invitrogen, Carlsbad, CA, USA). CYPA stable knockdown CAOV3 cells were screened by shRNA lentivirus infection and used for the in vivo metastasis assays.

### Quantitative PCR assay

Trizol reagent (#15596026, Invitrogen, Carlsbad, CA, USA) was used to extract total RNA from both CAOV3 and OVCAR3 cells. Then the total RNA was reverse-transcribed by M-MLV reverse transcriptase (M1701, Promega, Madison, Wisconsin, USA).

Total RNA was reversely transcribed to produce cDNA by cDNA synthesis system including dNTP, primer, 5 × PrimeScript buffers, DTT and DEPC water. Quantitative real-time PCR was performed using SYBR Ex Taq kit (#638319, Takara, Japan), and the relative expression level of CYPA was normalized to the expression of GAPDH.

### Immunoblot assays

Both SOC cells or tissues were lysed in RIPA Buffer (#9800, Cell Signaling, Danvers, MA) to extract proteins. Then the total protein samples was analyzed by SDS-PAGE. Subsequently the polyvinylidene fluoride (PVDF) membranes were blocked with 5% milk-TBST buffer and then incubated with the primary antibodies for the detection of CYPA, MMP3, MMP9, and β-actin for 1.5 h. Then the PVDF membranes were incubated with HRP-conjugate secondary antibodies for 1 h. Signals were visualizal with an ECL kit. Image Pro software was used in this assay to calculate the intensity of each blot.

### Cell motility assays

For wound closure assays, both CAOV3 and OVCAR3 cells were transfected with control or CYPA shRNA plasmids and grown as confluent monolayers. Then mechanically wound was made with a 20-L pipette tip to generate the wound. Cell debris was washed by PBS, and the culture medium was added to induce wound healing. Wound was photographed at 0 h and 20 h, and the extent percentage of wound closure was measured.

For transwell assays, CAOV3 and OVCAR3 cells were transfected with control or CYPA shRNA plasmids for 48 h and then trypsinized, re-suspended in serum-free medium. The upper chambers of Transwell filters (8.0 μm membrane pores) were subsequently coated with 20% matrigel and incubated at 37 °C for 30 min. A total of 10^5^ cells in 150 μl of medium were then added to the upper chambers of the inserts and were allowed to migrate toward the bottom chambers, which contained medium with 10% FBS. After 24 h, the remaining cells in the top chamber were removed, and cells on the underside were fixed in 4% paraformaldehyde and stained with 0.1% crystal violet for 30 min. Quantification of migrated cells was performed by dissolving crystal violet with 10% acetic acid, and the cell number of each sample was calculated.

### Tumor metastasis assays

All animal assay procedures were approved by our Institutional Animal Care and Use Committee. CAOV3 cells were stably transfected with control or CYPA shRNA lentivirus. About 5 × 10 ^5^ cells were implanted into the tail vein of athymic nude mice. After 8 weeks, the tumor was isolated, and weighted.

### Attention

We have done the Image splicing in Figs. 3 and 4.

### Statistics

Data were analyzed with SPSS 22.0 software and shown as the the mean ± standard deviation (SD) in vitro and in vivo assays. Student’ s t-test was used for statistical comparisons, and *P* < 0.05 is considered significant. The association between KIF3B expression and clinicopathological features was studied using the χ^2^ test.

## Results

### CYPA expression is correlated with the survival rate and clinical features of serous ovarian cancer

In decades, the involvement of CYPA in the progression of multiple cancers has been widely reported. To explore the potential function of CYPA in SOC development, we detected the expression level in SOC tissues of patients who underwent surgical resection performing IHC assays. Notably, the staining results revealed that CYPA was mainly located in the cytoplasm of SOC cells (Fig. 1a). We further explored and analyzed the difference of CYPA expression level between SOC tissues and adjacent tissues performing IHC assays. As expected, adjacent tissues showed obvious low expression level of CYPA compared with SOC tissues (Fig. 1a, b).

**Fig. 1:** CYPA was highly expressed in SOC tissues. **a** and **b** Immunohistochemistry assays were performed, and the representative photographs of CYPA expression level in SOC tissues were shown (× 100 and × 200 magnifications, respectively). **c** Immunohistochemistry staining showed the expression level of CYPA in adjacent tissues (× 100 and × 200 magnifications, respectively)

Based on the staining results, 82 tissue samples from SOC patients who underwent surgical resection were classified into low and high CYPA expression groups, according to the staining intensity (Fig. 1a and Table 1). According to the staining of tumor tissues, 42 patients showed low expression of CYPA, while 40 exhibited CYPA high expression (Table 1).

We further evaluated the clinical features of CYPA in patients with SOC. Patient age, tumor size, preoperative chemotherapy, tumor differentiation, FIGO stage, and lymphnode metastasis was analyzed, respectively. According to the analysis results, no obvious difference was found in clinical characteristics such as patient age and tumor grade between CYPA low and high expression groups (Table 1). Notably, our data revealed that CYPA expression was inversely associated with FITO stage (*p* = 0.040) and lymphnode metastasis (*p* = 0.015) in SOC patients (Table 1). In summary, these results indicated the possible involvement of CYPA in the progression of SOC.

### CYPA depletion impairs SOC cell migration and invasion in vitro

To evaluate the regulatory mechanism underlying CYPA affecting the progression of SOC, the shRNA specifically targeted CYPA was transfected into 2 types of human SOC cells, including CAOV3 and OVCAR3 cells, to inhibit the expression of CYPA. The results of quantitative RT-PCR assays (Fig. 2a) indicated that the transfection of CYPA shRNA plasmids effectively knock down its expression in both CAOV3 and OVCAR3 cells. Consistent with the results of quantitative RT-PCR assays, the immunoblot assays confirmed the obviously decreased expression levels of CYPA in both CAOV3 and OVCAR3 cells transfected with CYPA shRNA plasmids (Fig. 2b).

**Fig. 2:** CYPA expression was effectively inhibited in both CAOV3 and OVCAR3 human SOC cells after CYPA knockdown. **a** Quantitative RT-PCR assays revealed the obviously decreased expression level of CYPA caused by the transfection of its shRNA in CAOV3 and OVCAR3 cells, respectively. **b** Immunoblot assays confirmed the efficiently inhibition of CYPA expression after the transfection of CYPA shRNA plasmids in both CAOV3 and OVCAR3 cells. Results are presented as mean ± SD, * *P* < 0.05

We then performed wound healing and transwell assays to evaluate the effects of CYPA on the migration and invasion of SOC cells. Interestingly, our results revealed that knockdown of CYPA dramatically inhibited the extent of wound closure in both CAOV3 and OVCAR3 cells (Fig. 3a). In addition, CYPA knockdown significantly blocked the invasion of these 2 types of SOC cells through membranes, with dramatically dropped cell numbers (Fig. 3b). MMP3 and MMP9, which were generally known as markers of cells with high metastasis capacity, was detected in control and CYPA ablation groups. We found that the expression of MMP3 and MMP9 was reduced in CYPA shRNA-transfected CAOV3 and OVCAR3 cells, respectively (Fig. 3c, d).

**Fig. 3:** CYPA depletion prevents the migration and invasion of SOC cells in vitro. **a** Knockdown of CYPA led to the lower migration degree in CAOV3 and OVCAR3 cells. Photographs showing that at the 0, 20th hour time point migrated cells were present. **b** Transwell assays using both CAOV3 and OVCAR3 human SOC cells transfected with control or CYPA shRNA plasmids, and the degree of invasion was quantified by the invasion cell number. **c** Immunoblot assays showed the expression of MMP3 in control or CYPA shRNA-transfected CAOV3 and OVCAR3 cells, respectively. **d** Immunoblot assays revealed the expression level of MMP9 in control or CYPA depletion CAOV3 and OVCAR3 cells. Results are presented as mean ± SD, * *P* < 0.05. We have done the Image splicing in Fig. 3

Collectively, our results showed that CYPA promotes cell migration and invasion of SOC in vitro.

### CYPA induces the metastasis of SOC in vivo

Based on the previous results, CYPA ablation led to the inhibition of the migration and invasion of SOC cells, we further evaluated the possible function of CYPA in the metastasis of SOC in mice.

To confirm our hypothesis, we performed lung metastasis assay in mice. CAOV3 cells were infected with CYPA shRNA lentivirus to stably knockdown the expression of CYPA. Subsequently, control or CYPA depletion SOC cells injected into the caudal vein of nude mice. After 8 weeks, we found that the incidence of lung metastasis for CAOV3 cells was obviously reduced compared with the control groups (Fig. 4a).

**Fig. 4:** CYPA depletion inhibited the metastasis of SOC in mice. **a** CAOV3 cells infected with control or CYPA shRNA lentivirus were implanted into the caudal vein of nude mice. After 8 weeks, tumors were isolated and weighted . (*n* = 6 for each group). **b** IHC assays indicated the expression level of CYPA in control or CYPA knockdown tumor tissues isolated from mice. **c** IHC assays showed the difference of MMP3 expression level in tumor tissues isolated from control or CYPA depletion groups. **d** IHC assays showed the difference of MMP9 expression in tumor tissues isolated from different groups. Results are presented as mean ± SD, * P < 0.05. We have done the Image splicing in Fig. 4

To confirm the inhibition efficiency of CYPA expression in mice, we examined CAOV3 expression levels in tumor tissues through IHC assays. As was expected, we found that the expression level of CYPA in CYPA knockdown group was significantly reduced (Fig. 4b).

Furthermore, we examined the expression levels of MMP3 and MMP9 in tumor tissues from control and CYPA ablation groups by IHC assays. Consistent with our hypothesis, a significant dropped expression level of MMP3 and MMP9 was found in tumor tissues from knockdown groups, compared with control, suggesting the inhibition of migration capacity caused by CYPA ablation (Fig. 4c, d). In conclusion, our data indicated that CYPA was involved in the metastasis of SOC in mice.

## Discussion

Ovarian cancer is one of the hardest human malignancy in female reproductive organs with high metastasis [25]. The incidence rate of OC is second only to cervical cancer [26]. Among them, serous ovarian cancer (SOC) is one of the most malignant types [27]. For the treatment of SOC, traditional chemotherapy is difficult to achieve effective therapeutic effects [28]. Recently, a started multicentre randomized controlled trial about the cytoreductive surgery followed by chemotherapy versus chemotherapy alone for recurrent platinum-sensitive epithelial ovarian cancer, and the results proved that the therapy can improve progression free survival in selected patients with first recurrence of platinum-sensitive epithelial ovarian cancer [29]. Complete cytoreduction matched with adjuvant chemotherapy continues to be the effective therapy to be attempted in the surgical treatment of advanced ovarian cancer [30]. Accumulating evidence suggests that the management of ovarian cancer should be personalized taking into account the performance status of the patient, in particular in case of elderly women: The elderly patients can also benefit from standard treatment for ovarian cancer, but they are more fragile and with a lower life expectancy than the younger counterpart [31]. And more elderly patients were treated with neoadjuvant chemotherapy while less patients underwent surgery [32]. Because of the large and increasing number of elderly patients without treatment and the large survival gap, the opportunities for further improvements in the care for elderly ovarian cancer patients [32]. In fact, the progression free survival for patients diagnosed with advanced stage SOC is less than 18 months [2]. Therefore, targeted therapy and immunotherapy show broad prospects in the treatment of advanced SOC. Multiple genes were found highly expressed in recurrent SOC tissues such as SYK, AIF1, and WNK1, some of which were served as therapeutic targets for SOC treatment [9]. Interestingly, here we noticed CYPA was abnormal high expression in SOC tissues and involved in SOC progression, suggesting that it could be a novel therapeutic target of SOC.

CYPA, in a study, was reported as one of the malignant transformation-related proteins in esophageal cancer [33]. Additionally, CYPA was highly expressed in high metastatic melanoma compared with normal tissues [34]. Moreover, another study showed that CYPA was over-expressed in pancreatic cancer tissues, and the high expression of CYPA indicated high T stage and lymphnode metastasis [35]. Consistent with the results, in this study the high expression levels of CYPA were found in tumor tissues from patients with SOC. Interestingly, we analyzed the clinical features of SOC patients and found a significant link between clinical stage, lymphnode metastasis and CYPA expression. This clinical correlation also implies that CYPA plays an important role in the occurrence and metastasis of SOC.

To explore the possible role of CYPA in SOC development, the CYPA shRNA plasmids were transfected into 2 types of SOC cells: CAOV3 and OVCAR3 cells. Interestingly, we found that CYPA ablation dramatically blocked SOC cell migration and invasion by wound healing and migration assays in these 2 types of SOC cells. Additionally, immunoblot assays revealed that knockdown of CYPA reduced the expression levels of MMP3 and MMP9, suggesting that CYPA participates in the regulation of SOC metastasis. In fact, similar studies have been reported for other types of tumors. CYPA could promote the metastasis of non small cell lung cancer (NSCLS) through the p38/MAPK signaling pathway [21]. Several MMPs are regulated by p38/MAPK in multiple tissues such as bladder, skin, liver, and skin tissues [21]. Interestingly, we found the expression levels of 2 MMPs, MMP3 and MMP9, were obviously decreased caused by CYPA depletion in SOC cells, suggesting this process was possible regulated by p38/MAPK pathway. CYPA could bind prolactin and therefore promote the progression and metastasis of breast cancer [36]. These findings, together with our study, showed the critical role of CYPA on tumor metastasis. However, in pancreatic cancer, the in vitro results showed the effect of CYPA on the proliferation and apoptosis [35], which we could not find in this study (data not shown). Perhaps CYPA could play different roles in different types of tumors, and the precise mechanism underlying CYPA promoting the metastasis of different cancers was not clearly understood.

CYPA was first found as the target of cyclosporin A (CsA), an immunosuppressive drug, which has been used for the treatment of several tumors, including ovarian cancer [37]. Although the regulatory mechanism underlying CYPA promoting OC progression is still unclear, previous studies showed that CSA could bind to CYPA and thus increase the effects of chemotherapy [38]. In this research, we performed database analysis, in vitro and animal assays and found the potential link between CYPA expression and SOC progression. CYPA expression, similar to previous studies, was obviously correlated with clinical features of SOC patients, including tumor stage and lymphnode metastasis [33–38]. Our results are similar with previous studies indicating the important role of CYPA in tumorigenesis.

In several studies, CYPA was shown to regulate multiple gene expression by the physically interacting with transcription factors and histone modifying enzymes, and therefore affect various types of cellular processes [39, 40]. Since we found the role of CYPA in the metastasis of SOC, it was worth exploring the effects of transcription and histone modifying in SOC progression.

In summary, the current study reveals CYPA is highly expressed in SOC tissues, and correlated with the clinical features and prognosis of SOC patients. Further, CYPA promotes the metastasis of SOC both in vitro and in mice. These results help to provide a better understanding of the possible mechanisms of cancer progression and novel prognostic markers for SOC targeted therapy in the future.

## Data Availability

The raw data supporting the conclusions of this manuscript will be made available by the authors, without undue reservation, to any qualified researcher.
